# The Impact of Mixed-Ownership Reform on Innovation Performance of Manufacturing Companies: Evidence from China

This article has been retracted.

**DOI:** 10.1155/2022/3809829

**Published:** 2022-06-24

**Authors:** Wenlei Xia, Xiaofang Chen, Guangming Wang

**Affiliations:** ^1^School of Management, Wuhan University of Technology, Wuhan 430070, China; ^2^Research Institute of Digital Governance and Management Decision Innovation, Wuhan University of Technology, Wuhan 430070, China

## Abstract

Exploring the impact of a new round of mixed-ownership reform on enterprise development has far-reaching implications for the future development of mixed-ownership reform and the improvement of internal and external corporate governance of the enterprise. This study makes a comprehensive analysis of the relationship between mixed-ownership reform and innovation performance using a combination of empirical testing and theoretical analysis. In terms of theoretical analysis, this study summarizes research on mixed-ownership reform and innovation performance, while also integrating the theoretical basis of the development and institutional background of China's current mixed-ownership reform, and investigating the impact of mixed-ownership reform on innovation performance. A-share list of manufacturing companies from 2015 to 2018 is selected as the research object, and K-nearest neighbor matching, multiple regression model, and propensity score matching are used to test the effect of mixed-ownership reform on innovation performance. By comparing the changes in the innovation performance level of state-owned enterprises (SOEs) before and after the mixed-ownership reform, this study proposes that the SOEs will not only enhance the competitiveness among manufacturing companies but also will have a positive impact on the high-quality development of the entire society and industrial transformation and upgrading.

## 1. Introduction

Since the early 1990s, when the Chinese government chose to corporatize its state-owned firms, ownership reform has been at the center of the People's Republic of China's (PRC) economic reform program. The PRC's first Company Law was passed in 1993 to assist the fulfillment of this objective by creating a legal framework to renovate traditional SOEs (SOEs) into modern enterprises. SOEs reform has been implemented for about 40 years, starting with the introduction of township businesses as supplements, the separation of government and enterprises, the reform of the stock market system, and the ongoing mixed-ownership reform [1]. This is one of the most comprehensive and effective changes in the history of property rights ownership, resulting in increased efficiency in both production and resource distribution. It has the potential to become a focal point for economic growth and other academic studies. The mixed-ownership reform has now become the centerpiece of China's ongoing SOEs reform [2].

The construction of a modern Chinese economy is based on the real economy, with modern manufacturing and strategic emerging industries that reflect the progress of modern industries taking the lead, leading the future economic development [3]. As the micro-foundation and competitive main body of the market economy, enterprises are the most important part of the market main body and the most important force in the construction of a modern economic system [4]. Based on the classification reform, the reform of mixed ownership of SOEs has been promoted. The reform of SOEs is still trying to innovate and explore forward [5].

Scholars are now conducting an extensive study on the relationship between state-owned enterprise mixed reform and innovation [6]. Sun and Tong [7] evaluated the performance levels of 634 companies on the Shanghai and Shenzhen stock exchanges and found that state ownership has a negative impact on corporate performance. Chen et al. [8] studied Chinese listed companies and found that different types of companies have different owner efficiencies and SOEs have better efficiency. Lihui [9] examined 826 listed companies in China as research samples and reported that when the government shareholding ratio is lower than the threshold value, the company value decreases with the increase of government shareholding and increases with the increase of government shareholding, and the relationship between the two is “U-shaped.” Gompers et al. [10] examined US-listed companies and analyzed that the separation of two rights and corporate value showed a negative correlation. The author in [11] studied a list of companies in Indonesia and explored that the separation of two rights allows major shareholders to manipulate the company's earnings for their interests, resulting in the loss of corporate efficiency. Konijn et al. [12] focused on listed companies in the USA and determined that equity checks and balances are negatively related to enterprise value, and the negative impact is greater when the equity concentration is lower.

Various reform initiatives in the new wave of state-owned enterprise reform are substantially different from those in the past[13, 14]. Previously, enterprise property rights were frequently modified, and state-owned firms were directly transformed into private or other sorts of enterprises [15]. However, the present round of reforms focuses on introducing numerous types of property rights, which are reinforced by other reform initiatives and are no longer a single way of reform [16]. At the same time, the enterprise's external environment is considerably different from the past, requiring the application of new theories that conform to the current development trend [17].

Using a combination of empirical testing and theoretical research, this study explores the association between mixed-ownership change and innovation performance. In terms of theoretical analysis, this study highlights research on mixed-ownership reform and innovation performance and integrates the theoretical basis of the development and institutional background of China's current mixed-ownership reform. Moreover, the impacts of mixed-ownership reform on innovation performance are also investigated. In the empirical test, *K*-nearest neighbor matching, multiple regression model, and propensity score matching are used to test the effect of mixed-ownership reform on innovation performance. The outcomes of this study will help the management improvement of SOEs, to promote the development of SOEs, and provide assistance for the subsequent reform of SOEs.

The rest of the manuscript is organized as follows: Section 2 provides a background for mixed-ownership reforms in China.  Section 3 describes the impacts of SOEs mixed reform on innovation performance of manufacturing companies.  Section 4 describes different innovation tests, and section 5 concludes the manuscript.

## 2. Background

China's mixed-ownership reform is still in its early stages of development. The reform of mixed-ownership has been aided by the continuous development of the economy, the growing global environment, and the changing social structure [18]. Innovation performance is an important reflection of an enterprise's core competitiveness and competitive advantage [19]. Up to now, many scholars have carried out research on the measurement of enterprise innovation performance, the difference in innovation performance among enterprises with different property rights, and the influence of shareholders on enterprise innovation performance, and have produced certain conclusions and results. The existing literature believes that the nature of enterprise property rights will significantly affect the innovation performance of enterprises [20, 21]. In the long mileage of mixed-ownership reform, SOEs have improved their innovation performance and enhanced their competitiveness.  Figure 1 shows the impact path of mixed-ownership reform on innovation performance.

The primary reason for the lack of innovation power of SOEs is that there is an interest-dependent relationship between SOEs and local governments. Local governments depend on SOEs to transfer their policy burdens. SOEs rely on local governments to provide preferential policies to obtain high returns [22]. The larger the state-owned shareholding ratio of SOEs, the stronger the local government's dependence and control on SOEs, the more policy protection the SOEs receive, and the fewer external competitors. However, such characteristics do not meet the strategic needs of SOEs, so SOEs lack the motivation to use innovation to obtain external competitive advantages [23]. In addition, compared with the pursuit of profit maximization by non-SOEs, SOEs with both government and shareholder status pursue more maximization of social welfare, and different responsibility requirements make SOEs lack innovation motivation. SOEs have institutional problems such as unclear property rights, incomplete performance appraisal, and opaque executive appointments and removals, all of which will become restrictive factors for independent innovation [24]. Therefore, this study proposes the hypothesis that mixed-ownership reform can promote SOEs innovation. After the mixed-ownership reform, the reduction in the proportion of state-owned equity means that the political pressure exerted by the government on enterprises is reduced, which is conducive to the independent choice of enterprises to carry out more innovation activities [25]. Each investor can achieve economies of scale and specialized division of labor by integrating the resources of the enterprise to achieve complementary advantages and further increase the investment in R&D and the quality of product innovation, so as to improve the overall innovation capability of the enterprise. Secondly, the entry of nonstate-owned shareholders can enable enterprises to form a multi-equity structure with reasonable checks and balances, improve corporate governance, reduce the short-sighted behavior of management, and pay more attention to innovative activities that can bring long-term benefits to the enterprise [26, 27].

## 3. The Impact of SOEs Mixed Reform on Innovation Performance of Manufacturing Companies

### 3.1. Innovation Performance Evaluation Indicators

Independent innovation activities are very complex. Establishing a performance evaluation system for innovation activities is not only required but also useful for businesses. To avoid the short-board phenomena in the barrel principle, the evaluation of innovation performance evaluation indicators should reflect the company's innovative strength. In the innovation performance evaluation system, the selection of each indicator must be scientific, true, and accurate, and at the same time, it must be operable in practical applications. Therefore, it must be constructed based on rigorous, objective, comparable, and feasible benchmark innovative performance evaluation system. According to the above principles, this study examines the innovation performance level of enterprises from the aspects of innovation input and innovation output at the same time [28]. Moreover, in terms of innovation investment, this study refers to existing research and selects research and development (R&D) as a measurement factor for innovation investment. There are many R&D indicators to measure, including the ratio of innovation investment to operating income, a relative value such as R&D investment, and absolute value such as R&D investment. Because the research is carried out in the context of mixed-ownership reform, the income of enterprises may be manipulated, resulting in relatively large changes in the market value of enterprises, so the natural logarithm of R&D investment is used as a measurement factor. In terms of innovation output, the main selection criterion is the number of patents. Therefore, this study investigated the innovation output of enterprises from the perspective of patents, and the three patents of the utility model, design, and innovative invention are important indicators to measure patents. Therefore, the measure of innovation output in this study is assigned to the number of patent applications.

### 3.2. Data Sources and Sample Selection

This study selects the “Guidelines for the Industry Classification of Listed Companies” issued by the China Securities Regulatory Commission in 2012 as the standard for sample division and selects A-share listed manufacturing companies from 2015 to 2018 as the research object. The main reason for this selection is mainly because of the innovative nature of the research object, which is reflected in the manufacturing field. We selected the data source of the CSMAR database and the data that can be consulted on the Internet of listed companies in some samples. To ensure that the data can be presented completely and credibly, we processed the data as follows. First, we deleted the data samples of ST and ^*∗*^ST companies in the selected enterprises.  Table 1 defines the main variables.

Considering mixed-ownership reforms, SOEs are usually targeted. Therefore, the main object of analysis in this study is SOEs, so the data of nonstate-owned listed companies are excluded. In addition, based on the full-text description, two types of samples that fluctuate in the proportion of state-owned equity and show a clear upward trend are also excluded. In the end, 1,120 samples of data were included for innovation input, 720 samples of data were used for innovation output, and a total of 704 samples of data from the experimental group that had implemented mixed-ownership reform were named sample 1. At the same time, many companies will not be very active in applying for patents out of their interests. Therefore, when processing data, this study eliminated those companies that have never applied for patents or invention patents in the past 4 years. There are 472 samples of data in the experimental group (with mixed-ownership reform), and the above data are named sample 2. During the research process, the research on innovation input was used to sample 1, and the research on innovation output was used in sample 2, respectively.

### 3.3. Innovation Performance Evaluation Model

In this section, the *K*-nearest neighbor matching method is used to explore the differences in innovation performance between companies that implement mixed-ownership reform and companies that do not implement mixed-ownership reform. For the obtained data samples to perform propensity score matching, the main purpose is to find the control group, that is, the paired group of SOEs that have not implemented mixed-ownership reform and SOEs that have implemented mixed-ownership reform to form a counterfactual. Specifically, we name the experimental group (*T*) and the control group (C), and let *A* = {*T*, *C*} denote all samples. The matching method is to find similar enterprises that have not undergone mixed-ownership reform in the control group with a similar probability to the experimental group, to eliminate the selection bias. The model can be formulated as

(1) $$\begin{array}{c} P=\mathrm{Pr}\left\{A=T\right\}=\emptyset \left\{X_{i,t}\right\}, \end{array}$$

where *P* refers to the probability of mixed-ownership reform of enterprises, that is, the propensity score. Both groups of companies are paired based on this indicator, and *X(i,t)* is the matching variable. The indicators selected in this study mainly include the logarithm of total assets, the situation of two jobs concurrently, the asset-liability ratio, the operating net interest rate, and the return on total assets, respectively.

The K-nearest neighbor method is a very simple and effective classification method, which is widely used in pattern recognition. The starting point of the *K*-nearest neighbor method is to estimate the probability density function of the sample distribution. This method requires the function to be continuous and smooth so that the probability density function *p(x)* at point *x* can be estimated. Consider a very small field *R* surrounding *x* with volume *V*:

(2) $$\begin{array}{c} P\left(x\right)V=\int p\left(u\right)\text{d}u. \end{array}$$

In a field centered on the feature vector *x*, the fixed number of samples falling into the region *R* is *k(n).* Under a suitable distance scale, the volume of the region surrounding *x* is gradually increased until *k* sample points fall into this region. These are the *k(n)* samples around *x* that are closest to it. The probability density function estimate can be expressed as follows:

(3) $$\begin{array}{c} \hat{p}\left(x,n\right)\approx \frac{k\left(n\right)/n}{V\left(n\right)}. \end{array}$$

If the number of samples around *x* is small, the corresponding region will become large, and the volume *V(n)* of the region will also become large, so the resulting probability density value will become small. If the number of samples around *x* is large, the volume *V(n)* of the region will become small, so resulting in a large probability density value. The matching and identification method based on the k-nearest neighbor method is to take the *K*-nearest neighbors of the unknown sample *f*, and see which category most of the *K*-nearest neighbors belong to, and to which category *f* is classified. That is, in *N* known samples, find the *K*-nearest neighbors off.

## 4. Innovation Performance Test

### 4.1. Innovative Descriptive Statistics

For manufacturing SOEs, the difference in corporate investment between innovation input and innovation output is not very large, which shows that SOEs have been responding to and calling for the construction of an “innovative country” the state in recent years, and they have been improving its innovation performance level. This also shows that the core competitiveness of enterprises in the manufacturing industry is the innovation performance-level enterprises.  Table 2 presents descriptive results for all samples, whereas Table 3 describes the variable descriptive statistics of the reformed enterprise sample.

The difference between the asset-liability ratios of enterprises is obvious. The minimum value of the asset-liability ratio is 0.079, while the maximum value is 0.863. This shows that although both are SOEs, there are significant differences between enterprises. Well-run SOEs can maintain a good asset ratio, while poorly run SOEs face a higher risk of bankruptcy. The side shows the necessity of mixed-ownership reform. Only by implementing mixed-ownership reform can the decline of state-owned manufacturing enterprises, which have a key impact on development, be effectively reversed. In the overall sample, the proportion of SOEs that have implemented mixed-ownership reform is about 60%, which shows that the proportion of enterprises that have carried out mixed-ownership reform and the enterprises that have not carried out mixed-ownership reform selected in this study is about the same, and there is no such thing as one party overwhelming the other. Condition: The mean value of the time variable of mixed-ownership reform is 0.7. From these data, we can see that the selected sample from Chinese enterprises has more years after mixed-ownership reform than before reform.

### 4.2. Innovation Input/Output Matching Balance Test

The propensity score matching method is used to perform *K*-nearest neighbor matching and find similar SOEs that have not undergone mixed-ownership reform according to the weights assigned by propensity score matching. In the research sample from 2015 to 2018, the propensity score of each state-owned enterprise that has undergone mixed-ownership reform is calculated based on the observable matching variables, the corresponding SOEs were selected from the data that have not undergone mixed-ownership reform, and these SOEs form the control group. After the matching is completed, excluding the enterprises that have not been successfully matched, there are 172 enterprises that have undergone mixed-ownership reform (reform = 1) within the common value range, and a total of 102 enterprises that have not implemented mixed-ownership reform (reform = 0). Among them, 114 enterprises have undergone mixed-ownership reform with a complete number of patents, and 60 enterprises have not undergone mixed-ownership reform with a complete number of patents. The matching accuracy passed the verification requirements. The evaluation of innovation performance evaluation indicators should reflect the company's innovation strength, not only one aspect, to prevent the short-board phenomenon in the barrel principle. Therefore, this study examines the innovation output of enterprises from the perspective of patents, and the three patents of the utility model, design, and innovative invention are important indicators to measure patents in my country. There was no major difference between the two groups of data after matching, there was no major standardized deviation for the completely matched variables, and the matching deviation was less than 20%.  Table 4 describes the results of the innovation input matching balance test, and Table 5 shows the results of the innovation output matching balance test.

Tables 4 and 5 show that in terms of innovation input and output, enterprises that have not adopted mixed-ownership reform outperform enterprises that have implemented mixed-ownership reform. Before matching, there are significant differences in enterprise-scale, asset-liability ratio, operating net interest rate, and return on total assets. As a result, the number of patent applications is used as the measure of innovation output in this study. There are 472 samples of data in the experimental group (with mixed-ownership reform), and the above data are named sample 2. Sample 1 will be used in the study on innovation input, while sample 2 will be used in the research on innovation output. However, after matching, it can improve its insignificant degree, and the *T* value after matching is not significant, which shows that the general situation of the enterprises selected after matching is the same. After matching, the average treatment effect (ATT) of the treatment group with mixed-ownership reform and the control group without mixed-ownership reform is obtained.  Table 6 shows the estimated results.

As can be seen from Table 6, in terms of innovation input, the difference between the prereform and postreform is 0.597, which proves that the innovation input increases by 0.597% and the *T* value is 2.11 compared with the enterprises that have implemented the mixed-ownership reform. It shows that the average treatment effect (ATT) of the treatment group is significant at the 5% level; in terms of innovation output, the difference between prereform and postreform is 0.352%, which proves that compared with enterprises that have not yet implemented mixed-ownership reform, the innovation output increased by 0.352%, and the *T* value is 2.04, indicating the average.

Treatment effect (ATT) of the treatment group was significant at the 5% level. As a result, the hypothesis of this study is verified; that is, compared with companies without mixed-ownership reform, companies that have implemented mixed-ownership reform perform better in both innovation input and innovation output.

## 5. Conclusion

The construction of a modern economy is based on the real economy, with modern manufacturing and strategic emerging industries that reflect the progress of modern industries taking the lead, leading the future economic development of China. This study analyzes the relationship between mixed-ownership reform and innovation performance with the help of empirical testing and theoretical analysis. By comparing the changes in the innovation performance level of SOEs before and after the mixed-ownership reform, the effect of mixed-ownership reform policies was highlighted and the differences between the experimental group and the control group in many aspects (total assets, growth, financial leverage) affecting innovation capabilities of the two types of enterprises were examined. To avoid biasing the results of this work, one of the follow-up research aims is to add as many elements that impact the two types of organizations' innovation capacities into the model as much as possible. Future work will focus on expanding the sample to a larger market and joining the industry for consideration.

## Figures and Tables

**Figure 1:** The impact path of mixed-ownership reform on innovation performance.

**Table 1:** Variable definitions.

Type of variable	Variable name	Variable code	Variable meaning
Dependent variable (enterprise innovation performance evaluation index)	Innovation input	Lnrdspend	The logarithm of *R* & *D* investment
	Innovation output	Lnpatents	Add 1 to the number of patent applications in the year to take the natural logarithm

Independent variable	Mixed ownership reform	Reform	0 for unreformed firms and 1 for reformed firms
	Time variable	Time	0 before the reform, 1 after the reform

Control variable	Company size	Inside	Logarithm of total assets
	Financial leverage	Lev	Assets and liabilities
	Two-job situation	Dual	The combination of chairman and general manager takes 1; otherwise, it is 0.
	Market competition	Compete	Selling expenses/operating income
	The proportion of independent directors	Indratio	Number of independent directors/board size
	Return on assets	Roa	Return on total assets (net profit/total average assets)
	Operating net profit margin	Opr	Net profit/operating income
	Number of employees	Lnlabor	The natural logarithm of the number of employees
	Ownership concentration	Concern	The Herfindahl coefficient of the shareholding ratio of the largest shareholder
	Fixed asset investment	Rta	Net fixed assets/total assets
	Year	Year	Year of the company

**Table 2:** Variable descriptive statistics of all samples.

Variable	Observations	Average value	Standard deviation	Minimum	Maximum
Lnrdspend	1120	18.205.	1.343	14.214	22.060
Inpatents	720	2.718	1.289	0	5.760
Reform	1120	0.629	0.501	0	1
Lnsize	1120	23.478	1.126	20.190	26.893
Lev	1120	0.478	0.193	0.079	0.863
Dual	1120	0.664	0.472	0	0.368
Roe	1120	0.193	2.590	−0.452	0.329
Compete	1120	0.076	0.070	0.011	0.571
Indratio	1120	0.463	0.063	0.333	0.382
Roa	1120	0.030	0.107	−0.391	0.24
Opr	1120	0.086	0.243	−0.493	10.692
Lnlabor	1120	9.092	1.182	5.280	0.682
Concern	1120	0.269	0.153	0.014.	0.656
Rta	1120	0.365	0.178	0.091	22.060

**Table 3:** Descriptive statistics of variables in the sample of reformed enterprises.

Variable	Observations	Average value	Standard deviation	Minimum	Maximum
Lnrdspend	704	18.36	1.489	14.214	21.773
Lnpatents	472	2.44	1.452	0	4.780
Time	704	0.703	0.464	−5.760	0.992
Lnsize:	704	22.258	1.293	0.079	0.862.
Lev	704	0.476	0.201	−0.452	0.367
Dual	704	0.685	0.453	0.011	0.325
Roe	704	0.109	2.020	0.333	0.563
Compete	704	0.071	0.063	−0.376	0.382
Indratio	704	0.472	0.063	−0.493	0.22
Roa	704	0.028.	0.112	5.280	10.692
Opr	704	0.054	0.225	0.014	0.681.
Lnlabor	704	8.916	1.195	0.091	0.656.

**Table 4:** Innovation input matching balance test.

Mean						*T*-test	
Variable name	Deal with	Treatment group	Control group	Standard deviation (%)	Difference	*T* value	*P* > *T*
Lnsize	Before match	23.119	22.751	29.3	76.1	2.09	0.037
	After matching	23.119	23.207	−7.0		−0.38	0.701

Dual	Before match	0.93662	0.87069	22.4	100.0	1.82	0.070
	After matching	1	1	0.0		0.00.	1.000

Lev	Before match	0.47804	0.4489	15.1	79.6	1.21	0.226
	After matching	0.46696.	0.46101	3.1		0.15	0.881

Opr	Before match	0.05221	0.01781	28.2	75.3	2.24	0.026
	After matching	0.03239	0.04088	−7.0		−0.44	0.661

Roa	Before match	0.03657	0.02246.	25.6	98.8	2.01	0.045
	After matching	0.02646	0.02663	−0.3		−0.02	0.985

**Table 5:** Innovation output matching balance test.

Mean						*T*-test	
Variable name	Deal with	Treatment group	Control group	Standard deviation (%)	Difference	*T* value	*P* > *T*
Lnsize	Before match	22.444	21.826	68.0	99.5	5.15	0.000
	After matching	22.444	22.447	−0.4		−0.02	0.984

Dual	Before match	0.92308	0.63008	75.0	99.5	4.85	0.000
	After matching	0.92308	0.92462	−0.4		−0.03.	0.974

Lev	Before match	0.4694	0.34977	69.8	92.0	5.54	0.000
	After matching	0.4694	0.45979	5.6		0.34	0.737

Opr	Before match	0.05604	0.09669	−36.7	79.0	−2.52	0.012
	After matching	0.05604	0.04748	7.7		0.32	0.752

Roa	Before match	0.03787	0.05036	−23.1	69.9	0.31	0.109
	After matching	0.03787	0.03412	−6.9.		5.15	0.755

**Table 6:** Estimated results.

Variable name	Sample	Treatment group	Control group	Difference	Standard deviation	*T* value
Lnrdspend	After matching (ATT)	18.343	17.746	0.597	0.282	2.11
Lnpatents	After matching (ATT)	4.697	4.345	0.352	0.172	2.04

## Data Availability

The data required for this study are already included in the article.
